The article "Influence of antidepressants on plasma levels of nitric oxide metabolites in patients with major depressive disorder" was retracted in 2022. Reasons: errors in the analysis; errors in the methods; concerns about the data.

# Influence of antidepressants on plasma levels of nitric oxide metabolites in patients with major depressive disorder

**DOI:** 10.1192/bjo.2021.1074

**Published:** 2021-12-17

**Authors:** Atsuko Ikenouchi, Naomichi Okamoto, Yusuke Konno, Rintaro Fujii, Yoshihisa Fujino, Reiji Yoshimura

**Affiliations:** Department of Psychiatry, School of Medicine, University of Occupational and Environmental Health, Japan; and Medical Center for Dementia, University Hospital, University of Occupational and Environmental Health, Japan; Department of Psychiatry, School of Medicine, University of Occupational and Environmental Health, Japan; and Medical Center for Dementia, University Hospital, University of Occupational and Environmental Health, Japan; Department of Psychiatry, School of Medicine, University of Occupational and Environmental Health, Japan; Department of Psychiatry, School of Medicine, University of Occupational and Environmental Health, Japan; Department of Environmental Epidemiology, Institute of Industrial Ecological Sciences, University of Occupational and Environmental Health, Japan; Department of Psychiatry, School of Medicine, University of Occupational and Environmental Health, Japan

**Keywords:** Depression, nitric oxide, antidepressants, norepinephrine, cardiovascular disease

## Abstract

The impairment of endothelial function by reduced endothelial production of nitric oxide (NO) may contribute to the increased risk of developing cardiovascular disease in patients with depression. NO also plays an essential role in the efficacy of antidepressants. The present study aimed to confirm our previous preliminary findings using a larger sample and different antidepressants. We enrolled 100 patients with major depressive disorder (MDD) and 50 healthy controls. Patients were administered sertraline, duloxetine or mirtazapine and were followed up for 8 weeks. We also compared the rate of increase in plasma levels of metabolites of NO (NOx) among the three antidepressant treatments. Baseline plasma NOx levels were significantly lower in the MDD group than in the control group. A negative correlation was found between plasma NOx levels and the severity of MDD. Treatment with duloxetine significantly increased plasma NOx levels, whereas sertraline treatment caused no significant increase.

Physically healthy patients with depression have an increased risk of developing cardiovascular disease (CVD).^1^ A meta-analysis of prospective cohort studies found that major depressive disorder (MDD) was associated with a significantly increased risk of myocardial infarction and coronary death.^2^ This association indicates that endothelial dysfunction may be involved in the development of depression.

The article "Influence of antidepressants on plasma levels of nitric oxide metabolites in patients with major depressive disorder" was retracted in 2022. Reasons: errors in the analysis; errors in the methods; concerns about the data.

Nitric oxide (NO) is a small free radical that plays a critical signalling role in physiology and pathophysiology. Producing sufficient amounts of NO to regulate vascular resistance and maintain adequate blood flow is important for healthy functioning of the vascular system. Endothelial nitric oxide synthase (eNOS) is a constitutive NOS form in endothelial cells that contributes significantly to vascular NO levels under physiological conditions.^3^ Since NO can be rapidly inactivated by haemoglobin or oxidised to forms of nitrogen dioxide such as nitrates and nitrites (NOx), the plasma NOx level is often used as an indicator of NO production in blood vessels.^4^ eNOS immunoreactivity decreased in a rat model of depression.^5^ The possible role of NO in depression has been confirmed through the link between an increased risk of coronary heart disease and NO production, and the effects of antidepressants on NO production.^6–8^ We previously reported that milnacipran, a serotonin–noradrenaline reuptake inhibitor, increased plasma levels of NOx in patients with MDD using a small sample.^9^ The present study aimed to confirm our previous preliminary findings using a larger sample and different antidepressants.

## Method

### Participants

This study included 100 Japanese in-patients and out-patients who met DMS-IV-TR criteria^10^ for a first episode of MDD without psychotic features and who scored 8 or higher on the 17-item Hamilton Rating Scale for Depression (HRSD-17).^11^ We also enrolled 50 gender- and age-matched healthy controls recruited from a group of Japanese healthcare workers. We screened for illness history using a questionnaire. All the patients were physically healthy, had no history of psychiatric disorders and had not used any psychotropic medications in the past 6 months; they had not taken antidepressants or mood stabilisers for at least 2 weeks prior to the start of the study. All the patients and healthy controls were non-smokers with no history of CVD.

All participants initially underwent electrocardiography and blood tests to rule out cardiovascular and hepatic dysfunction. Severity of depression was evaluated using the HRSD-17. During this study the patients were treated with the antidepressants sertraline, duloxetine or mirtazapine (24, 48 and 28 patients, respectively) and followed for 8 weeks after initiation of treatment. The attending physician determined the type and dosage of antidepressant using a flexible dose design.

The authors assert that all procedures contributing to this work comply with the ethical standards of the relevant national and institutional committees on human experimentation and with the Helsinki Declaration of 1975, as revised in 2008. All procedures involving human patients were approved by the Ethics Committee of the University of Occupational and Environmental Health of Japan (Approval No. 09–08). Written informed consent was obtained from all participants.

The article "Influence of antidepressants on plasma levels of nitric oxide metabolites in patients with major depressive disorder" was retracted in 2022. Reasons: errors in the analysis; errors in the methods; concerns about the data.

### Blood samples and assay method

All blood samples were taken at 07.00 h before breakfast (at least 12 h after the last dose of medication). We obtained venous blood samples from participants while they were in a supine position. The plasma samples were separated in a centrifuge and stored at −80°C until analysis. Plasma NOx levels were analysed by the Griess method using high-performance liquid chromatography (ENO-20; Eicom, Kyoto, Japan).

### Statistical analyses

The clinical and biochemical data of the study participants are expressed as mean (s.d.). The association between HRSD-17 scores and plasma NOx levels was examined using Spearman's correlation coefficient. Differences in NOx levels between baseline and week 8 were examined by Wilcoxon matched-pairs signed-rank test as the plasma NOx levels were not normally distributed in the Kolmogorov–Smirnov test. The changes in plasma NOx levels in the antidepressant groups were compared using the Kruskal–Wallis test. This comparison was also undertaken using analysis of covariance to adjust for gender and age.

We conducted all statistical analyses using Stata 17 (Stata Corp LLC, College Station, Texas, USA). The statistical significance was set at *P* < 0.05.

## Results

Table 1 shows the characteristics of the study population. The HRSD-17 scores of the MDD group significantly decreased from baseline to 8 weeks after treatment with antidepressants. The plasma NOx levels at baseline were significantly lower in the MDD group compared with the control group (*P* < 0.001, *P-*adjusted for age and gender) and increased after 8 weeks of treatment. There was a negative correlation between the baseline HRSD-17 scores and plasma NOx levels (*r* = −0.278, *P* = 0.017), and between the HRSD-17 scores (week 8 – baseline) and NOx levels (week 8 – baseline) in patients with MDD (*r* = −0.269, *P* = 0.021).

**Table 1:** Characteristics of the study and control populations

	Control participants	Patients with major depressive disorders			
		Total	Antidepressant administered		
			Sertraline	Duloxetine	Mirtazapine
Participants, *n*	50	100	24	48	28
Gender, males/females	23/27	47/53	9/15	28/20	10/18
Age, years: mean (s.d.)	54 (7.1)	52.3 (16.1)	56.4 (15.4)	50.5 (15.8)	52.0 (17.1)
HRSD-17 at baseline, mean (s.d.)	−	19.4 (5.9)	22.0 (5.4)	18.0 (6.6)	19.3 (4.4)
HRSD-17 at week 8, mean (s.d.)	−	8.5 (5.1)	9.1 (6.3)	8.7 (4.4)	7.4 (5.0)
Plasma NOx level at baseline, mean (s.d.) (μM)	29.6 (1.7)	17.2 (9.3)	21.5 (10.5)	16.8 (8.0)	14.0 (9.3)
Plasma NOx level at week 8, mean (s.d.) (μM)	−	21.2 (13.5)	21.7 (12.5)	21.9 (12.1)	19.7 (16.9)
Difference in plasma NOx levels at baseline and week 8					
Mean (s.e.) (μM)		4.07 (1.45)	0.22 (2.89)	5.06 (2.05)	5.68 (2.90)
*P*-value^a^		0.0088	0.7751	0.0127	0.0451

HRSD-17, 17-item Hamilton Rating Scale for Depression; NOx, metabolites of nitric oxide.

a. The *P*-values are derived from Wilcoxon matched-pairs signed-rank test.

The article "Influence of antidepressants on plasma levels of nitric oxide metabolites in patients with major depressive disorder" was retracted in 2022. Reasons: errors in the analysis; errors in the methods; concerns about the data.

Eight weeks of treatment using duloxetine resulted in significantly increased plasma NOx levels (*P* = 0.0127). Sertraline and mirtazapine did not significantly change these levels. The changes in plasma NOx levels did not differ among the antidepressant groups (*P* = 0.1945). The results were similar for gender- and age-adjusted analysis of covariance (*P* = 0.224).

## Discussion

### Main findings

This study's findings showed that the plasma NOx levels of patients with MDD were significantly lower than those of healthy controls. Treating the depression with antidepressants recovered the plasma NOx levels. There was a negative correlation between the HRSD-17 score and plasma NOx concentration, confirming our preliminary findings.^9^ In contrast, in a study by Suzuki et al, the plasma NOx levels in patients with MDD were reported to be significantly higher than those in healthy controls and to decrease after recovery from MDD.^12^ Furthermore, there are several reports that suicide attempts in patients with mood disorders and schizophrenia are associated with elevated plasma NOx levels.^7,13^ Thus, the effect of plasma NOx levels on patients with MDD remains controversial.

Treatment with duloxetine, but not sertraline and mirtazapine, increased plasma NOx levels at week 8. We previously reported that in patients with MDD, administration of milnacipran, but not paroxetine, increased plasma NOx levels.^9^ Taking these findings into account, it is possible that duloxetine, which influences both serotonin transporters and noradrenaline transporters, increases plasma NOx levels. In contrast, paroxetine and sertraline both specifically only affect serotonin transporters and do not change plasma NOx levels. Seya et al demonstrated that norepinephrine induces eNOS activity.^14^ Graves & Poston also reported that NO is released from the endothelium of rat mesenteric resistance arteries by activation of β1-adrenergic receptors.^15^ Thus, antidepressants that influence norepinephrine neurons might play a role in affecting plasma NOx levels, mainly via noradrenergic signalling.

### Limitations

This study has some limitations. First, only plasma NOx levels were measured, and not eNOS activity. Second, body weight and body mass index, which influence plasma NOx levels, were not adjusted for. Third, plasma NOx levels in the control group were not assessed after 8 weeks. Fourth, and perhaps most importantly, a small sample size and weak statistical power may have influenced the outcome. Moreover, we used a flexible drug design. Therefore, further studies without these limitations need to be performed to obtain robust results.

The article "Influence of antidepressants on plasma levels of nitric oxide metabolites in patients with major depressive disorder" was retracted in 2022. Reasons: errors in the analysis; errors in the methods; concerns about the data.

In conclusion, NO might be partially involved in the pathophysiology of MDD, and some antidepressants affecting both noradrenaline and serotonin neurons increase plasma NOx levels in patients with MDD.

## Data Availability

The data that support the findings of this study are available on request from the corresponding author, A.I.

## References

[1] Lichtman JH, Bigger JT Jr, Blumenthal JA, Frasure-Smith N, Kaufmann PG, Lespérance F, Depression and coronary heart disease: recommendations for screening, referral, and treatment: a science advisory from the American Heart Association Prevention Committee of the Council on Cardiovascular Nursing, Council on Clinical Cardiology, Council on Epidemiology and Prevention, and Interdisciplinary Council on Quality of Care and Outcomes Research: endorsed by the American Psychiatric Association. Circulation 2008; 118: 1768–75.1882464010.1161/CIRCULATIONAHA.108.190769

[2] Wu Q, Kling JM. Depression and the risk of myocardial infarction and coronary death: a meta-analysis of prospective cohort studies. Medicine 2016; 95: e2815.2687185210.1097/MD.0000000000002815PMC4753948

[3] Huang PL, Huang Z, Mashimo H, Bloch KD, Moskowitz MA, Bevan JA, Hypertension in mice lacking the gene for endothelial nitric oxide synthase. Nature 1995; 377: 239–42.754578710.1038/377239a0

[4] Archer S. Measurement of nitric oxide in biological models. FASEB J 1993; 7: 349–60.844041110.1096/fasebj.7.2.8440411

[5] Demirtaş T, Utkan T, Karson A, Yazır Y, Bayramgürler D, Gacar N. The link between unpredictable chronic mild stress model for depression and vascular inflammation? Inflammation 2014; 37: 1432–8.2461494410.1007/s10753-014-9867-4

[6] Finkel MS, Laghrissi-Thode F, Pollock BG, Rong J. Paroxetine is a novel nitric oxide synthase inhibitor. Psychopharmacol Bull 1996; 32: 653–8.8993087

[7] Lara N, Archer SL, Baker GB, Le Mellédo JM. Paroxetine-induced increase in metabolic end products of nitric oxide. J Clin Psychopharmacol 2003; 23: 408–12.1292041910.1097/01.jcp.0000085416.08426.1d

[8] Rajagopalan S, Brook R, Rubenfire M, Pitt E, Young E, Pitt B. Abnormal brachial artery flow-mediated vasodilation in young adults with major depression. Am J Cardiol 2001; 88: 196–8.1144842510.1016/s0002-9149(01)01623-x

The article "Influence of antidepressants on plasma levels of nitric oxide metabolites in patients with major depressive disorder" was retracted in 2022. Reasons: errors in the analysis; errors in the methods; concerns about the data.

[9] Ikenouchi-Sugita A, Yoshimura R, Hori H, Umene-Nakano W, Ueda N, Nakamura J. Effects of antidepressants on plasma metabolites of nitric oxide in major depressive disorder: comparison between milnacipran and paroxetine. Prog Neuropsychopharmacol Biol Psychiatry 2009; 33: 1451–3.1966467610.1016/j.pnpbp.2009.07.028

[10] First MB, Spitzer RL, Gibbon M, Williams J. Structured Clinical Interview for DSM-IV-TR Axis I Disorders, Research Version. Biometrics Research, New York State Psychiatric Institute, 2002.

[11] Zimmerman M, Martinez J, Attiullah N, Friedman M, Toba C, Boerescu DA, Further evidence that the cutoff to define remission on the 17-item Hamilton Depression Rating Scale should be lowered. Depress Anxiety 2012; 29: 159–65.2249594210.1002/da.20870

[12] Suzuki E, Yagi G, Nakaki T, Kanba S, Asai M. Elevated plasma nitrate levels in depressive states. J Affect Disord 2001; 63: 221–4.1124609910.1016/s0165-0327(00)00164-6

[13] Kim YK, Paik JW, Lee SW, Yoon D, Han C, Lee BH. Increased plasma nitric oxide level associated with suicide attempt in depressive patients. Prog Neuropsychopharmacol Biol Psychiatry 2006; 30: 1091–6.1672524710.1016/j.pnpbp.2006.04.008

[14] Seya Y, Fukuda T, Isobe K, Kawakami Y, Takekoshi K. Effect of norepinephrine on RhoA, MAP kinase, proliferation and VEGF expression in human umbilical vein endothelial cells. Eur J Pharmacol 2006; 553: 54–60.1707051610.1016/j.ejphar.2006.09.048

[15] Graves J, Poston L. Beta-adrenoceptor agonist mediated relaxation of rat isolated resistance arteries: a role for the endothelium and nitric oxide. Br J Pharmacol 1993; 108: 631–7.809678110.1111/j.1476-5381.1993.tb12853.xPMC1908020

